The article "Classification of Resting-State Status Based on Sample Entropy and Power Spectrum of Electroencephalography (EEG)" was retracted in 2023. Reasons: signs of a paper mill; suspected computer-generated content; unreliable results or conclusions; lack of ethics approval or compliance.

# Classification of Resting-State Status Based on Sample Entropy and Power Spectrum of Electroencephalography (EEG)

**DOI:** 10.1155/2020/8853238

**Published:** 2020-11-10

**Authors:** Ahmed M. A. Mohamed, Osman N. Uçan, Oğuz Bayat, Adil Deniz Duru

**Affiliations:** ^1^School of Engineering and Natural Sciences, Altinbas University, 34217, Turkey; ^2^Department of Computer Science, The Libyan Academy, 16063 Benghazi, Libya; ^3^Faculty of Sport Science, Marmara University, 34668, Turkey

## Abstract

An electroencephalogram (EEG) is a significant source of diagnosing brain issues. It is also a mediator between the external world and the brain, especially in the case of any mental illness; however, it has been widely used to monitor the dynamics of the brain in healthy subjects. This paper discusses the resting state of the brain with eyes open (EO) and eyes closed (EC) by using sixteen channels by the use of conventional frequency bands and entropy of the EEG signal. The Fast Fourier Transform (FFT) and sample entropy (SE) of each sensor are computed as methods of feature extraction. Six classifiers, including logistic regression (LR), K-Nearest Neighbors (KNN), linear discriminant (LD), decision tree (DT), support vector machine (SVM), and Gaussian Naive Bayes (GNB) are used to discriminate the resting states of the brain based on the extracted features. EEG data were epoched with one-second-length windows, and they were used to compute the features to classify EO and EC conditions. Results showed that the LR and SVM classifiers had the highest average classification accuracy (97%). Accuracies of LD, KNN, and DT were 95%, 93%, and 92%, respectively. GNB gained the least accuracy (86%) when conventional frequency bands were used. On the other hand, when SE was used, the average accuracies of SVM, LD, LR, GNB, KNN, and DT algorithms were 92% 90%, 89%, 89%, 86%, and 86%, respectively.

## 1. Introduction

The electrical activities of the brain can be used to identify the mental state of a person. Additionally, brain health can be monitored by electrical signals, which can be noninvasively measured from the scalp surface. Several sensors can be attached to the scalp surface, and the electrical activity of the brain can be investigated using electroencephalography (EEG). Since the number of sensors (electrodes) is limited (1-256), the spatial resolution of the measured EEG is low when compared with the other brain activity measurement techniques. On the other hand, the temporal resolution of the EEG is in milliseconds. Among the brain imaging techniques, none of the methods can work at such a high temporal sensitivity except magnetoencephalography (MEG) which is not as practical as EEG. The electrical activities of the brain are projected through the scalp surface because their impulses pass through the skull, which filters the data acting as a low-pass filter. Thus, the scalp EEG should be carefully analyzed and processed to find out the mental state of the subject. For instance, the resting state of the brain can be assessed through the ongoing EEG measurements. To identify the resting state, EEG measurement is taken for a few seconds and power spectral analysis is performed. Signal processing is widely used to extract relevant information, which is hidden in the measured EEG signals. EEG data classification is used to identify the mental diseases in emotion recognition and mental state determination using a brain-computer interface (BCI) as well as through the monitoring of mental workload. The basic state that can be identified from the scalp measurements is the resting state of the brain when eyes are open or closed [1]. The identifiers of these two states are hidden in the frequency content of the measured signal; however, this identifier may also vary in groups of subjects [2].

The article "Classification of Resting-State Status Based on Sample Entropy and Power Spectrum of Electroencephalography (EEG)" was retracted in 2023. Reasons: signs of a paper mill; suspected computer-generated content; unreliable results or conclusions; lack of ethics approval or compliance.

### 1.1. Aim of the study

We aimed to identify the brain's resting status using short-length EEG epochs using both linear and nonlinear features derived from EEG. Conventional EEG band power values are generally linear, while sample entropy has been measured as complexity metrics of the multivariate signal. The concept behind this study is to adopt machine learning techniques, which are used for feature classification. Logistic regression (LR), K-Nearest Neighborhood (KNN), linear discriminant (LD), decision tree (DT) classifier, support vector machine (SVM), and Gaussian Naive Bayes (GNB) algorithms are implemented and evaluated when these techniques are performed with precision.

## 2. Literature Review

When the alpha band power of a depressed group of participants was compared to a normal group, low alpha band power was observed in both conditions (EC and EO) [3]. In a recent study, connectivity metrics of frontal and centro-parietal lobes were formed to classify the cases into EO and EC and the obtained accuracy values were high [4]. The same condition was studied based on wavelet fuzzy approximate entropy (WFAPEN) feature values based on support vector machine (SVM), and they reported an accuracy value of 88.2% [5]. Several studies have been conducted to analyze machine learning methodologies as a part of EEG classification. For instance, a new proposed model was applied to detect the case of vigilance or drowsiness for fast train drivers. In that study, the Fast Fourier Transform (FFT) was used to extract the power spectrum density (PSD) of EEG. They achieved 90.70% accuracy using SVM [6]. According to Saghafi et al. in [7], changing eye states EC and EO without any notice can affect the brain signals. They applied logistic regression (LR), support vector machine (SVM), and artificial neural network (ANN) classifiers. Their highest obtained accuracy was 88.2% for ANN, which detects the eye change in less than two seconds. Stepwise linear discriminant analysis (SWLDA) and Fisher's linear discriminant (FLD) showed the best performance because they were applied as parts of two kinds of methods, which were linear and nonlinear, to compare the classification techniques for the P300 Speller [8]. In a prediction study of the eye states, while using EEG signals, stacked autoencoders (SAE) and deep belief network (DBN) classifiers were used with 98.9% accuracy for the designed SAE models [9]. An effective technique was introduced that can be implemented to identify sleep stages using new statistical features, which are applied to individual EEG signals for 10-second epoch durations [10]. The distance computation like Manhattan, Minkowski, Euclidean, Hamming, and Chebyshev can affect the accuracy of a classifier. Isa et al. in [11], showed 70.08% KNN accuracy as the highest classification with Minkowski distance computation. Two classified conditions, which are represented in positive and negative emotions collected by EEGÖzerdem and Polat in [12], indicated 77.14% accuracy for multilayer perceptron neural network (MLPNN) and 72.92% for K-Nearest Neighborhood (KNN). Based on linear and nonlinear features derived from EEG, cognitive activity and resting-state conditions were classified by applying SVM and 92.1% was achieved applying nonlinear features whereas 87.5% of SVM was observed applying linear features [13].

The article "Classification of Resting-State Status Based on Sample Entropy and Power Spectrum of Electroencephalography (EEG)" was retracted in 2023. Reasons: signs of a paper mill; suspected computer-generated content; unreliable results or conclusions; lack of ethics approval or compliance.

## 3. Materials and Methods

### 3.1. Data Collection

Nine subjects participated during the resting-state EEG measurements. 16 electrodes (F3, Fp1, P3, O1, C3, FZ, T7, CZ, Fp2, F4, C4, T8, PZ, P4, O2, and OZ) were placed on the scalp surfaces of the participants using an active electrode cap with a V-amp device. The sampling rate was set at 1 kHz. Subjects were asked to close their eyes without focusing on an idea for 3 minutes while their brain signals were being collected using EEG. Then, the other 3 minutes of measurement was taken while the eyes were in an open condition. According to studies of functional resting-state magnetic resonance imaging (rs-fMRI), the keeping choice of EC and EO tasks in the resting-state studies is considered a critical factor that has a series of effects on the brain activity patterns [14, 15]. The detection of neural mechanisms of various diseases has been widely used by rs-fMRI [16] because it is suitable for patients who are unable to cooperate and respond to the task paradigms [17]. Figures 1–3, respectively, show the signals for different durations, the first second, the half-second, and the end time second of recording signals from one subject in the case of close eyes.

Figures 4–6 show the signals in the time of the first second, the half-second, and the end time second of recording signals from the same subject in the case of open eyes.

### 3.2. Preprocessing and Feature Extraction

For further analysis, the absolute amplitude of epochs which is greater than 100 *μ*V was removed additionally, this study requires feature extraction, for which, the Fast Fourier Transform and sample entropy were used along with logistic regression (LR) classifier, K-Nearest Neighbor (KNN), linear discriminant (LD) analysis, decision tree (DT) classifier, support vector machine (SVM), and Gaussian Naïve Bayes (GNB) algorithms, which were used for classification purposes. Figures 7 and 8 show the power spectrum as an example of extracted features for closed and open eyes, respectively.

Fourier Transform (FT) is used to transform time-domain measurements into the frequency domain. FT divides the function into a continuous band called the spectrum of frequencies [18]. Fast Fourier Transform (FFT) is an algorithm that computes the FT at a fast pace [19].

The general formula of the Fast Fourier Transform is shown in Eq. (1).

(1) $$\begin{array}{c} X\left(k\right)=\overset{N-1}{\underset{n=0}{\sum }}x\left[n\right]w_{N}^{kn}=\underset{n\text{even}}{\sum }x\left(n\right)w_{N}^{kn}+\underset{n\text{odd}}{\sum }x\left(n\right)w_{N}^{kn},k=0,1,\cdots \cdots ,N-1, \end{array}$$

where *X*(*k*) represents the Fourier coefficients of *x*(*n*), which is assumed to have a complex value (sample of the time series, which consists of *N* samples), even *n* and odd *n* correspond to the even-numbered and odd-numbered samples of *x*(*n*), for frequency *k*, respectively. Here, *w* = exp(−2*πj*/*N*), and *j* = √−1; hence, *j* can be considered as an imaginary unit.

The second method used for feature extraction in this study was the sample entropy (SE). It is used to measure the complexity and regularity of time series [20]. The general formula of sample entropy is shown in Eq. (2).

(2) $$\begin{array}{c} H\left(R\right)=-\overset{n}{\underset{i=1}{\sum }}\text{p}\text{i}\log2\left(\text{pi}\right), \end{array}$$

where *R* is a random variable that takes on values from the set {R1, R2, . . ., Rn} with respective probabilities p1, p2, . . ., pi, where ∑*i*pi = 1. Then, the entropy of *R*, *H*(*R*), represents the average amount of information contained in *R*, and pi is a proportion of samples that belongs to class *n* for a particular node.

The article "Classification of Resting-State Status Based on Sample Entropy and Power Spectrum of Electroencephalography (EEG)" was retracted in 2023. Reasons: signs of a paper mill; suspected computer-generated content; unreliable results or conclusions; lack of ethics approval or compliance.

### 3.3. Classification

For classification, K-Nearest Neighbor (KNN) was implemented as a first step, which was presented in the early 1950s, and it works with the enormous datasets for pattern recognition. Classifiers of the nearest neighbor depend on the comparison of similarity between training tuples with a given test tuple that represents an analogy learning step between them. This method works by using an n-dimensional pattern space, and the training tuples are put into it. KNN works as the density evaluator to distribute the training data. Based on the extracted features, which are also considered as training patterns, the data can be classified by applying KNN [21]. By Euclidean distance formula, this distance can be determined; the formula of Euclidean distance is shown below in Eq. (3).

(3) $$\begin{array}{c} \text{dis}\left(\text{x}1,\text{x}2\right)=\overset{n}{\underset{i=1}{\sum }}\sqrt{{\left(\text{x}1\text{i}-\text{x}2\text{i}\right)}^{2}}, \end{array}$$

where x1 refers to tuple x1, x2 refers to tuple 2, and x11, x12,……, x1i express the number of features in tuple 1, whereas x21, x22,……,x2i represent the number of features in tuple 2.

The second method that has been used for analysis in this paper is logistic regression. It is a statistical method that deals with two kinds of classes. Also, logistic regression helps to make predictions, and it is used to develop a regression model based on a categorically dependent variable. It deals with the variable vector that evaluates the input variable coefficients [22]. Respectively, the regression model is defined by Eqs. (4) and (5).

(4) $$\begin{array}{c} z=a_{0}+\overset{n}{\underset{i=1}{\sum }}a_{i}x_{i}, \end{array}$$

(5) $$\begin{array}{c} P\left(z\right)=\frac{e^{z}}{1+e^{z}}, \end{array}$$

where *z* is the contribution measure of the explanatory variables; the regression coefficients can be represented by *x*_*i*_(*i* = 1 ⋯ *n*), *a*_*i*_, which were obtained by maximum likelihood in conjunction with their standard errors represented in *∆a*_*i*_ and*P*(*z*).

Logistic regression has three types: (I) binary, which deals with a variable response as a binary response; (II) multinomial that has more than two unordered sets; (III) ordinal that has ordered sets.

The next classifier was the decision tree (DT) that works on huge stored data and transforms the data into helpful knowledge. DT is considered as a tree, and this tree has internal nodes (non leaf node) while each of them expresses a test based on an attribute, and the outcome of the test acts as a branch and a class label holed by each end node (leaf node) [23]. The process of DT learning from a class-labelled training data tuples is known as induction of DT. Attribute selection measures like information Gain and Gini index are used during tree construction to select the attributes that best partition data tuples into distinct classes. Gini index measures the impurity of data *D* from a set of training tuples as written in Eq. (6).

(6) $$\begin{array}{c} \text{Gini}\left(D\right)=1-\overset{m}{\underset{i=1}{\sum }}\text{p}{\text{i}}^{2}, \end{array}$$

where pi represents the probability of a tuple in *D* belonging to a class Ci and can be estimated using ∣Ci, *D* | /∣*D*∣.

The article "Classification of Resting-State Status Based on Sample Entropy and Power Spectrum of Electroencephalography (EEG)" was retracted in 2023. Reasons: signs of a paper mill; suspected computer-generated content; unreliable results or conclusions; lack of ethics approval or compliance.

Information gain is a measure that finds the attribute with the highest information gain which helps to minimize the information required to classify a data tuple. Information gain is defined as in Eq. (7).

(7) $$\begin{array}{c} \text{Info}\left(D\right)=-\overset{m}{\underset{i=1}{\sum }}\text{p}{\text{i}}^{2}\log_{2}\text{pi}, \end{array}$$

where pi is the probability that a tuple in dataset *D* could belong to a specific class, say Ci.

Linear discriminant analysis is a method of alleviation of linear dimensions. It is used to identify the linear features, which increase the separation between classes of data and reduce the scattering within a class [24]. The classifier of LDA is used to estimate both mean and variance of the entered data using a function, which is given below in Eq. (8).

(8) $$\begin{array}{c} \mu =\frac{1}{nk}\sum x. \end{array}$$

For the class (*k*), (*n*) is the total number of observations and *μ* represents the mean of the input (*x*).

By using Eq. (9), variance is computed for all the model inputs.

(9) $$\begin{array}{c} \sigma^{2}=\frac{1}{n-k}\sum {\left(x-\mu \right)}^{2}, \end{array}$$

where *σ*^2^ represents the variance of all the inputs of the model.

The Naive Bayes method is known as a supervised classification algorithm, which does not need a huge amount of data for training. Naive Bayes classifiers perform very fast. With a normal distribution and big data, the Gaussian process can generate them [22, 25, 26], as shown in Eq. (10).

(10) $$\begin{array}{c} p\left(x_{i}/y\right)=\frac{1}{\sqrt{2\pi \sigma_{y}^{2}}}\exp\left(-\frac{{\left(x_{i}-\mu_{y}\right)}^{2}}{2\pi \sigma_{y}^{2}}\right), \end{array}$$

where parameters *σ*_*y*_ and *μ*_*y*_ are estimated by maximum likelihood.

The last classifier used in this paper is the support vector machine (SVM), which is a classification method for linear and nonlinear datasets. SVM provides a learning model by separating between separable classes through constructing a hyperplane. The goal is to find the hyperplane that best separates and provides the highest distance margin between points of data tuple [26, 27]. Let *W* be the data vector normal to hyperplane and *b* the displacement of that vector; then, the decision function *D* for input *z* can be defined by Eq. (11).

(11) $$\begin{array}{c} D\left(z\right)=W∙z-b, \end{array}$$

where $z\in \left\{\begin{array}{cc} A & \text{if}D\left(z\right)>0\\ B & \text{if}D\left(z\right)<0 \end{array}\right.$.

The article "Classification of Resting-State Status Based on Sample Entropy and Power Spectrum of Electroencephalography (EEG)" was retracted in 2023. Reasons: signs of a paper mill; suspected computer-generated content; unreliable results or conclusions; lack of ethics approval or compliance.

The distance from *z* to the hyperplane is defined by Eq. (12).

(12) $$\begin{array}{c} \frac{D\left(z\right)}{\;|\;\left|W\right|\;|\;}. \end{array}$$

### 3.4. Confusion Matrix

The confusion matrix evaluation has been applied in the current study. The classification is quantifiable using the confusion matrix. According to Han et al. in [28], classifier analysis can be applied to recognize different classes with the help of confusion matrix tools. The performance matrix can be expressed in terms of confusion matrix using options such as true negative (TN), true positive (TP), false negative (FN), and false positive (FP).

*True negatives (TNs)*: they are correctly labelled negative records. TNs represent the number of true negatives.

*True positives (TPs)*: it classifies positive tuples that have been accurately labelled. TPs represent the number of true positives.

*False negatives (FNs)*: they are mainly positive records mislabelled as negatives, for instance, in our case study; the class with open eyes was wrongly predicted as the one with closed eyes by the classifier. FNs represent the number of false negatives.

*False positives (FPs)*: they are negative records that are incorrectly labelled “positive,” such as a record of class with closed eyes while the classifier prediction was open eyes. FPs represent the number of false positives. “Davis and Goadrich in [29]” described the confusion matrix, which is illustrated in Table 1.

Besides the mentioned ones, there are some other confusion matrix concepts such as “precision and recall”, which are commonly applied as classification methods. Recall measures completeness while precision measures exactness. Precision implies the real records' percentage, which is labelled “positive”. Recall implies the records' percentage, which is also labelled “positive”. Other ways of using precision and recall are to convert them into a single measure, which is termed as F1 score/F measure. Precision, recall, and F1 score considered as evaluation parameters. They can be computed by, respectively, using Eqs. (13), (14), and (15).

(13) $$\begin{array}{c} \text{Precision}=\frac{\text{TP}}{\text{TP}+\text{FP}}, \end{array}$$

where TP is a true positive and FP is a false positive.

(14) $$\begin{array}{c} \text{Recall}=\frac{\text{TP}}{\text{TP}+\text{FN}}, \end{array}$$

where TP is a true positive and FN is a false negative.

(15) $$\begin{array}{c} \text{F}1-\text{score}=\frac{2*\text{precision}*\text{recall}}{\text{Precision}+\text{recall}}. \end{array}$$

The sequence of this work is shown in Figure 9

The article "Classification of Resting-State Status Based on Sample Entropy and Power Spectrum of Electroencephalography (EEG)" was retracted in 2023. Reasons: signs of a paper mill; suspected computer-generated content; unreliable results or conclusions; lack of ethics approval or compliance.

## 4. Results

The results are presented in the following forms: average accuracy of classification/confusion matrix/parameter evaluation represented in precision, recall, and F1-score. The average accuracy value of the individual subjects, which was obtained from the features deduced by FFT, was the highest one (97%), which were obtained using LR and SVM algorithms. The accuracies achieved from the LD, KNN, and DT were 95%, 93%, and 92%, respectively. The minimum accuracy was computed for GNB (86%). Additionally, the average accuracy value of the individual subjects, which were obtained from the features extracted by SE, was 92% for SVM, 90% for LD, 89% for LR and GNB, and 86% for KNN and DT algorithms.

Tables 2 and 3 respectively show the accuracies of classifiers, confusion matrix, and parameter evaluation applied to the extracted features by FFT.

Tables 4 and 5 respectively show the accuracies of classifiers, confusion matrix, and parameter evaluation applied to the extracted features by SE.

## 5. Discussion

EEG played a significant role in several studies because its functions are based on pure brain signals. Using these signals, a lot of information can be obtained, specifically when this information is processed through cleaning, filtering, and sorting. It was noticed that different studies used different kinds of EEG. Besides, the numbers of electrodes, which can be 1, 4, 16, or even up to 256, record the signals directly from the brain tissue as an invasive technique or just from the scalp. Besides, EEG can be measured under different planned conditions, such as eyes closed, eyes open, or during the implementation of a cognitive task from healthy participants or patients [30]. In the concept of this study, we adopted three-minute measurements of EC and EO tasks as the resting-state paradigm.

Some studies were conducted to compare the accuracy when they twice used the SVM classifier with linear and nonlinear features. Moreover, the eyes' open condition was sustained for five minutes, during which, measurement signals were obtained from 128 electrodes in [13]. Other studies focused on the comparison between the results used in different algorithms. For instance, a comparative analysis was conducted to compare SVM and ANN to detect the events of eyes, such as closed, open, and blinking eyes. The highest accuracy was assured in the case of SVM [31]. The results of previous studies showed that the accuracy of the algorithms varied, depending on the different conditions they were operating with. In some of the EEG classification studies, varying accuracy values were reported as a result of different classifiers. However, in our study, similar accuracy values were achieved as in [32]. In EC and EO tests, the number of electrodes in our study was different compared to the ones used in previous studies and volunteers of our study showed a very high degree of compliance with the instructions given to them. The execution time of classification algorithms was less than a minute in the present study. Some different factors that can affect the results of a lot of studies represented in the numbers of electrodes of EEG, the length of windows, number of subjects who may be healthy or patients' volunteers, the ways of feature extraction, the stimulus which can be used, numbers of classifiers, and so on. For instance, according to Zhang et al. in [6], there were ten participants and they used eight electrodes, whereas in our study, there were nine participants and we used sixteen channels. In [12], the number of channels of the EEG was thirty-two with twenty participants whereas our data came from sixteen channels. According to Ahmad et al. in [13], the number of channels was 128 with eight healthy participants. Djemal et al. [33] used two public datasets of a BCI competition, which was provided by Graz University represented in dataset IIa with nine participants and dataset IV with three participants. According to Duru in [34], the states of EO, EC, and increased mental workload MW were tried to be identified using the scalp of EEG measurements epoched with a duration of a second. Hence, the different factors can affect the result from such a study to another.  Table 6 shows the different results of different objective studies, which are comparable to our study.

The article "Classification of Resting-State Status Based on Sample Entropy and Power Spectrum of Electroencephalography (EEG)" was retracted in 2023. Reasons: signs of a paper mill; suspected computer-generated content; unreliable results or conclusions; lack of ethics approval or compliance.

From a BCI approach, the speed of the information extraction rate depends on the length of the EEG time series. Thus, when compared with the other studies, it can be observed that we can classify the two states using shorter time series, with similar accuracy values.

We achieved consistent accuracy values based on the usage of either FFT-based features or the SE features. The former feature set represents the oscillations in the time series while the latter mimics the regularity of the fluctuations. Finally, the response of the brain to the EC or EO stimuli can be discriminated by the computation of the features (by FFT or by SE) even from a one-second time period.

## Figures and Tables

**Figure 1:** Time series for a subject in the first second when the subject closed the eyes.

**Figure 2:** Time series for half second when eyes of the subject were close.

**Figure 3:** Time series for subject at the end time seconds in the case of close eyes.

**Figure 4:** Time series for subject during the first second with open eyes.

**Figure 5:** Time series for subject at the half seconds in the case of open eyes.

**Figure 6:** Time series for subject at the end time seconds in the case of open eyes.

**Figure 7:** Power spectrum in the case of close eyes. Different colors denote different EEG channels.

**Figure 8:** Power spectrum in the case of open eyes.

**Figure 9:** Sequential steps of our study.

**Table 1:** Confusion matrix.

	Actual positive	Actual negative
Predicted positive	TP	FP
Predicted negative	FN	TN

**Table 2:** Classification accuracies of classifiers applied to extracted features by FFT.

Subjects	KNN	LR	DT	LD	GNB	SVM
1	0.97	0.99	0.99	0.98	0.97	0.99
2	0.92	0.97	0.85	0.97	0.71	0.98
3	0.70	0.77	0.73	0.75	0.71	0.82
4	0.88	0.97	0.84	0.92	0.89	0.94
5	0.99	1.00	0.97	0.99	0.63	1.00
6	1.00	1.00	0.97	0.99	0.99	1.00
7	1.00	1.00	0.99	1.00	0.98	0.98
8	0.96	1.00	1.00	1.00	0.99	0.99
9	0.99	0.99	0.97	0.99	0.90	0.99
Average accuracy	0.93	0.97	0.92	0.95	0.86	0.97

**Table 3:** Confusion matrix and parameter evaluation of classifiers applied to extracted features by FFT.

Classifiers	Confusion matrix			Parameter evaluation		
KNN		Close	Open	Precision	Recall	F1-score
	Close	35	1	0.92	0.97	0.94
	Open	3	34	0.96	0.91	0.93
LR		Close	Open	Precision	Recall	F1-score
	Close	36	1	0.97	0.97	0.97
	Open	1	36	0.97	0.97	0.97
DT		Close	Open	Precision	Recall	F1-score
	Close	34	3	0.94	0.92	0.94
	Open	2	35	0.92	0.95	0.93
LD		Close	Open	Precision	Recall	F1-score
	Close	36	1	0.97	0.97	0.97
	Open	1	36	0.97	0.97	0.97
GNB		Close	Open	Precision	Recall	F1-score
	Close	35	1	0.84	0.97	0.89
	Open	9	28	0.95	0.76	0.82
SVM		Close	Open	Precision	Recall	F1-score
	Close	35	1	0.97	0.97	0.96
	Open	3	34	0.97	0.97	0.97

**Table 4:** Classification accuracies of classifiers applied to extracted features by SE.

Subjects	KNN	LR	DT	LD	GNB	SVM
1	0.71	0.77	0.72	0.78	0.72	0.82
2	0.88	0.93	0.89	0.93	0.93	0.96
3	0.83	0.88	0.87	0.87	0.89	0.92
4	0.79	0.81	0.70	0.81	0.71	0.77
5	0.85	0.90	0.90	0.92	0.96	0.96
6	0.99	0.99	0.96	0.99	0.98	0.99
7	0.94	0.97	0.95	0.97	0.98	0.98
8	0.87	0.87	0.90	0.89	0.91	0.93
9	0.92	0.93	0.89	0.92	0.93	0.97
Average accuracy	0.86	0.89	0.86	0.90	0.89	0.92

**Table 5:** Confusion matrix and parameter evaluation of classifiers applied to extracted features by SE.

Classifiers	Confusion matrix			Parameter evaluation		
KNN		Close	Open	Precision	Recall	F1-score
	Close	90	2	0.82	0.97	0.89
	Open	22	69	0.96	0.77	0.85
LR		Close	Open	Precision	Recall	F1-score
	Close	83	9	0.89	0.90	0.89
	Open	10	81	0.90	0.89	0.89
DT		Close	Open	Precision	Recall	F1-score
	Close	79	13	0.89	0.86	0.86
	Open	11	80	0.86	0.89	0.87
LD		Close	Open	Precision	Recall	F1-score
	Close	85	8	0.89	0.92	0.90
	Open	11	80	0.92	0.88	0.90
GNB		Close	Open	Precision	Recall	F1-score
	Close	84	8	0.90	0.91	0.90
	Open	10	81	0.90	0.89	0.89
SVM		Close	Open	Precision	Recall	F1-score
	Close	87	5	0.92	0.94	0.93
	Open	9	82	0.94	0.91	0.92

The article "Classification of Resting-State Status Based on Sample Entropy and Power Spectrum of Electroencephalography (EEG)" was retracted in 2023. Reasons: signs of a paper mill; suspected computer-generated content; unreliable results or conclusions; lack of ethics approval or compliance.

**Table 6:** Different results of different objective studies compared with our study.

Researchers	Objectives of study	Algorithms used	Accuracy (%)
[6]	They proposed a fatigue detection system based on monitoring high-speed train drivers by wireless EEG.	SVM	90.70
[12]	Classification for positive and negative emotions used in the EEG signals.	MLPNN KNN	77.14 72.92
[13]	Classifying the resting states of the human brain using linear and nonlinear EEG features	SVM with non-linear features SVM with linear features.	92.1 87.5
[33]	Improving the three-class motor imagery (MI) with BCI classification accuracy	LDA SFFS	86.06 93
[34]	Imposing to increase the mental workload (mw)	Average accuracies of KNN, SVM, and DT	94, 88, 89
[35]	Effectiveness of the discrete wavelet transform (DWT) in load recognitions signatures	KNN, SVM DT, RF Adaboost, GBoosting GaussianNB, LDA QDA	98.93, 64.93 100, 95.33 61.20, 100 66.53, 69.06 19.06
Present work	Identifying the resting-state status of brain using short-length EEG epochs	Extracted features by FFT: KNN, LR, DT, LD, GNB, SVM Extracted features by SE: KNN, LR, DT LD, GNB, SVM	93, 97, 92, 95, 86, 97 86, 89, 86 90, 89, 92

## Data Availability

The data used for this study are available from the corresponding authors, [AMAM and ADD], upon reasonable request.
